# Loquat Leaf Extract Enhances Muscle Contraction-Induced Activation of Protein Synthesis Signaling in Rat Skeletal Muscle

**DOI:** 10.1155/2022/2234118

**Published:** 2022-06-24

**Authors:** Yung-Li Hung, Riki Kosugi, Toshiharu Natsume, Shuichi Machida

**Affiliations:** ^1^Institute of Health and Sports and Medicine, Juntendo University, 1-1 Hirakagakuendai, Inzai, Chiba 270-1695, Japan; ^2^Faculty of Health and Sports Science, Juntendo University, 1-1 Hirakagakuendai, Inzai, Chiba 270-1695, Japan; ^3^COI Project Center, Juntendo University, 2-1-1 Hongo, Bunkyo, Tokyo 113-8421, Japan; ^4^Graduate School of Health and Sports Science, Juntendo University, 1-1 Hirakagakuendai, Inzai, Chiba 270-1695, Japan

## Abstract

Loquat (*Eriobotrya japonica* (Thunb.) Lindl.) leaves are traditionally used to improve muscle weakness, but their effects on muscle protein synthesis require further research. Therefore, we aimed to investigate whether loquat leaf extract (LLE) enhances muscle contraction-induced activation of muscle protein synthesis signaling. Male Wistar rats (12 weeks old, *n* = 6/group) were categorized into water treatment (CON) and LLE treatment (LLE) groups. The rats were administered distilled water or LLE (1.5 g/kg/day) once a day by oral gavage for 7 days. On day 7, at 3 h post-LLE administration, the gastrocnemius muscle in the right leg of each rat was stimulated by electrical muscle stimulation (EMS) (100 Hz, 30 V) through five sets of 10 isometric contractions (7 s contraction, 3 s rest) with 3 min interset intervals. The rats were then sacrificed, and the gastrocnemius muscles of both legs were excised at 3 h post-EMS. The phosphorylation levels of mammalian target of rapamycin complex 1 (mTORC1) signaling pathway molecules (Akt, mTOR, and p70S6K) were determined by Western blotting. Regarding the muscle contraction-induced protein synthesis signaling pathway, Akt phosphorylation at Ser473 was not significantly different between the CON and LLE groups. mTOR phosphorylation at Ser2448 was increased by EMS but did not show a significant difference between the CON and LLE groups. p70S6K phosphorylation at Thr389 was significantly increased in response to EMS, whereas the LLE group showed significantly higher p70S6K phosphorylation at Thr389 than that in the CON group. This suggests that LLE enhances muscle contraction-induced activation of p70S6K phosphorylation in rat skeletal muscles.

## 1. Introduction

Skeletal muscle constitutes approximately 40% of human bodyweight; it is a key component of daily physical activity and contributes to the quality of life. Skeletal muscle mass and strength decrease because of aging and disease [1]. Severe loss of skeletal muscle mass and strength, as in sarcopenia and chronic kidney disease-related muscle wasting, leads to reduced mobility [2]. Maintaining skeletal muscle mass for normal physical activity and quality of life in patients with such diseases is rather challenging. In this context, therapeutic strategies for maintaining or increasing muscle mass are important for preserving mobility in later years.

Mammalian target of rapamycin complex 1 (mTORC1) is a key regulatory factor in the initiation of mRNA translation and is known to regulate skeletal muscle protein synthesis and subsequent muscle hypertrophy [3]. The upstream components of the mTORC1 pathway are involved in phosphoinositide 3-kinase (PI3K)/Akt signaling. The 70 kDa ribosomal protein S6 kinase (p70S6K), which plays an important role in mRNA translation initiation, is a key downstream target of mTORC1. Thus, mTORC1 signaling (Atk-mTOR-p70S6K) is thought to be involved in mTORC1 activity and subsequent muscle protein synthesis [4].

Several traditional herbal medicines, such as Go-sha-jinki-Gan, *Astragalus* polysaccharides, and *Astragali radix*, show potential therapeutic effects in sarcopenia and disease-related muscle wasting [5–7]. However, clinical trials on the use of traditional herbal medicines in treating sarcopenia and disease-related muscle wasting remain lacking and require further investigation in future. Loquat (*Eriobotrya japonica* (Thunb.) Lindl.) leaves have been used as traditional herbal medicine in several countries to treat cough and nausea [8, 9]. Loquat leaf extract (LLE) has been shown to effectively protect against aging-induced skeletal muscle loss [10]. Furthermore, a previous study has shown that LLE supplements inhibit dexamethasone-induced reduction in muscle strength in Sprague-Dawley rats [11]. Overall, these results suggest the possibility of using LLE as a therapeutic agent to prevent skeletal muscle atrophy. Enhancing muscle protein synthesis and reducing muscle breakdown are important treatment options for muscle weakness. However, the effects of LLE on muscle protein synthesis remain unknown.

Resistance exercises improve skeletal muscle mass by muscle protein synthesis via the mTORC1 signaling pathway [12]. A previous study has demonstrated that LLE enhances mTORC1 signaling (Akt-mTOR-p70S6K) [10]. A combination of balanced nutrition and exercise is considered an effective strategy for increasing muscle mass. We thus hypothesized that LLE stimulates mTORC1 signaling and enhances mTORC1 signaling in combination with resistance exercise. To test our hypothesis, we investigated the effects of LLE alone and in combination with resistance exercise on the mTORC1 signaling pathway in rat skeletal muscles. Overall, the aim of this study was to investigate whether LLE enhances muscle contraction-induced activation of protein synthesis signaling.

## 2. Materials and Methods

### 2.1. Loquat Leaf Extraction

Dried loquat leaves (China, HB60511) were purchased from Uchidawakanyaku (Tokyo, Japan). LLE was prepared as previously described, with modifications [7, 11]. Twenty grams of LLE was crushed into a powder, soaked in 200 ml distilled water at 23 ± 1°C for 30 min, and boiled at low heat for 30 min. The decoction was passed through a mesh filter and centrifuged at 4000 rpm for 12 min at 23 ± 1°C. The supernatant was filtered and stored at −80°C until use. The LLE concentration was approximately 0.25 g/ml. High-performance liquid chromatography (HPLC) showed that the amount of ursolic acid (UA) was 7.16 mg/100 mL of LLE and 0.4 mg/kg bodyweight/day.

### 2.2. Animal Experiments

The study protocol was approved by the Juntendo University Animal Care Committee (19-07). A previously described electrical muscle stimulation (EMS)-induced muscle contraction protocol was followed [13] with some modifications. Twelve male Wistar rats (12 weeks old) were divided into two groups and administered either LLE or distilled water following a week of acclimation. The rats were purchased from Japan SLC, Inc. (Shizuoka, Japan) and housed under controlled environmental conditions (23 ± 1°C, 55 ± 5% relative humidity) under a 12 h light/dark cycle with ad libitum access to water and a standard laboratory diet. The rats were administered LLE (1.5 g/kg/day) [11] or distilled water intragastrically by oral gavage using feeding needles (Fuchigami Kikai, Kyoto, Japan) under light isoflurane anesthesia, once a day for 7 days. All groups were starved for 12 h prior to the seventh day of administration. On day 7, 3 h after administration, the rats were anesthetized in an induction chamber with 3.0% isoflurane mixed with 21% O_2_ and 78% N_2_. The hair on the right lower hind limb was shaved and removed using a depilatory cream. Each anesthetized rat was then placed prone in a cradle specifically designed for stimulating the right gastrocnemius muscle. Throughout a typical experiment, anesthesia was maintained by gas inhalation through a facemask that continuously supplied 2.0% isoflurane mixed with 21% O_2_ and 78% N_2_, using an open-circuit gas anesthesia machine. One electrode was placed at the knee joint, and the other was placed at the heel. The foot was fixed to the pedal at 90° to stretch the right gastrocnemius muscle. The electrical stimulator was used to discharge monophasic rectangular pulses. The gastrocnemius muscle of the right leg of the rats was subjected to EMS (100 Hz, 30 V) through five sets of 10 isometric contractions (7 s contraction, 3 s rest) with 3 min interset intervals. The rats were sacrificed by heart removal, and gastrocnemius muscles were collected 3 h after EMS. The gastrocnemius muscles of both legs were obtained the from rats in the water treatment (CON) and LLE treatment (LLE) groups (*n* = 6/group).

### 2.3. Western Blot Analysis

The gastrocnemius muscles were frozen and powdered in liquid nitrogen followed by homogenization in T-PER Tissue Protein Extraction Reagent (Thermo Scientific, Waltham, MA, USA) containing protease (Thermo Scientific) and phosphatase inhibitors (Roche, Basel, Switzerland). Protein concentration was measured using the BCA protein assay reagent according to the manufacturer's instructions (Thermo Scientific). Muscle protein extracts (20 *μ*g) were separated by electrophoresis on a 10% SDS polyacrylamide gel and electroblotted onto PVDF membranes. The membranes were incubated with 5% skim milk in Tris-buffered saline/Tween 20 (TBST) for 1 h at 23 ± 1°C, followed by overnight incubation with primary antibodies at 4°C. All antibodies were purchased from Cell Signaling Technology (Danvers, MA, USA), including phospho-Akt Ser473 (cat. no. 4060), total Akt (cat. no. 4691), phospho-mTOR Ser2448 (cat. no. 5536), total mTOR (cat. no. 2983), phospho-p70S6K Thr389 (cat. no. 9234), and total p70S6K (cat. no. 2708). Blots were washed thrice with TBST and incubated with a horseradish peroxidase-conjugated secondary antibody (1 : 5000 dilution) for 1 h at 23 ± 1°C. Blots were again washed thrice with TBST and developed using an ECL chemiluminescence substrate (Amersham, Buckinghamshire, UK). Band intensities were quantified using the Image Lab v.5.2.1 software (Bio-Rad Laboratories, Hercules, CA, USA). The blots were then stained with Ponceau S to verify equal protein loading.

### 2.4. Statistical Analysis

All data are expressed as mean ± standard deviation (SD). Statistical analysis was performed using two-way ANOVA followed by Tukey's post hoc test using the GraphPad Prism 5 software (San Diego, CA, USA). Statistical significance was set at *p* < 0.05.

## 3. Results and Discussion

### 3.1. Bodyweight, Water Intake, and Diet Intake

Bodyweight, water intake, and diet intake were not significantly different between the LLE and distilled water groups after 7 days (data not shown).

### 3.2. Muscle Contraction-Induced Muscle Protein Synthesis Signaling

Regarding muscle contraction-induced mTORC1 (Akt-mTOR-p70S6K) signaling, Akt phosphorylation at Ser473 was not affected in response to EMS (Figure 1). mTOR phosphorylation at Ser2448 increased in response to EMS, but was not significantly different between the CON and LLE groups (Figure 2). p70S6K phosphorylation at Thr389 was significantly increased in response to EMS, whereas the LLE group showed significantly higher p70S6K phosphorylation at Thr389 compared with the CON group (Figure 3).

## 4. Discussion

In the present study, we investigated the effects of loquat (*Eriobotrya japonica* (Thunb.) Lindl.) leaf extract on muscle contraction-induced activation of protein synthesis signaling. Our results indicate that LLE administration alone did not affect mTORC1 signaling, but it enhanced muscle contraction-induced mTORC1 signaling via activation of p70S6K phosphorylation at Thr389 in rat skeletal muscles. These findings suggest that the effect of LLE administration on mTORC1 signaling was not additive, but synergistic with muscle contraction. On the other hand, our results demonstrate that LLE administration dramatically increased p70S6K phosphorylation at Thr389, but did not significantly change Akt phosphorylation at Ser473 compared with that in the control group. In a previous study, Akt phosphorylation (Ser473) was affected by LLE treatment in vitro [10]. Thus, the effects of LLE may differ between in vitro and in vivo settings.

Previous studies have demonstrated a relationship between mTOR/p70S6K and muscle protein synthesis. Ogasawara and Suginohara reported that promotion of muscle protein synthesis by resistance exercise (transcutaneous electrical stimulation to induce muscle contraction) was regulated by mTOR (both rapamycin-sensitive mTORC1 and rapamycin-insensitive mTORC1 or mTORC2) [14]. However, a recent study reported that exercise-induced protein synthesis is independent of mTOR/p70S6K. You et al. reported that protein synthesis by mechanical loading is mTORC1-independent in myotenectomy-induced muscle hypertrophy [15]. Different experimental methods for inducing muscle hypertrophy-like electrical stimulation or myotenectomy-induced muscle hypertrophy may also result in different pathways of muscle protein synthesis. Therefore, the relationship between mTOR/p70S6K expression and muscle protein synthesis remains unclear. We did not elucidate the relationship between mTOR/p70S6K and muscle protein synthesis induced by EMS in this study either. However, the EMS-induced increase in muscle protein synthesis is regulated by mTOR/p70S6K signaling [14].

Figueiredo et al. demonstrated that mTOR Ser2448 is part of a negative feedback loop mechanism involving p70S6K phosphorylation [16]. However, mTOR Ser2448 phosphorylation has been shown to induce muscle contraction-induced activation of mTORC1 and p70S6K phosphorylation in previous studies [17, 18]. Furthermore, suppression of Akt Ser473 phosphorylation was found to reduce p70S6K Thr389 phosphorylation in a previous study [19]. Taken together, the findings demonstrate that phosphorylation of Akt Ser473, mTOR Ser2448, and p70S6K Thr389 is activated by muscle contraction and plays central roles in muscle contraction-induced muscle protein synthesis.

Many active compounds, including UA, have been identified in LLE. An in vivo study showed that UA reduces muscle atrophy and stimulated hypertrophy [20]. Furthermore, UA enhances p70S6K phosphorylation at Thr389 but does not affect Akt phosphorylation at Ser473 in response to resistance exercise [21]. In contrast, chronic administration of UA (6 weeks) was found to affect Akt phosphorylation in a previous study [22]. However, a single administration of UA did not affect Akt phosphorylation (ser473) [21]. Thus, the effect of LLE may differ between single and chronic administrations. These findings are consistent with those of the present study. Here, we investigated the effects of LLE on mTORC1 signaling at 3 h after muscle contraction. Ogasawara et al.indicated that UA enhanced p70S6K phosphorylation at Thr389 6 h after resistance exercise, but did not affect Akt phosphorylation at Ser473 [21]. The main effect of UA on the muscle contraction-induced mTORC1 signaling is thought to occur via p70S6K. Our results suggest that LLE augments mTORC1 signaling through activation of p70S6K at Thr389. However, further studies are needed to determine the optimal time point for contraction-induced protein synthesis after muscle contraction following LLE administration.

This study has some limitations. First, we assessed only one time point after muscle contraction. Second, the examined protein synthesis signaling pathway was only limited to the mTORC1 (Akt-mTOR-p70S6K) signaling pathway. Thus, it did not examine the upstream components of the mTORC1 pathway, which are known to be involved in Akt and extracellular signal-regulated kinase 1/2 (ERK1/2) signaling [23], and the downstream targets of mTORC1, including eukaryotic initiation factor 4E-binding protein 1 (4E-BP1) and p70S6K, both of which play important roles in mRNA translation initiation. Third, muscle protein synthesis was not assessed in this study. These limitations need to be addressed in future studies.

## 5. Conclusions

Overall, our results indicate that LLE enhances muscle contraction-induced activation of p70S6K phosphorylation at Thr389 in rat skeletal muscles.

## Figures and Tables

**Figure 1:** Effects of LLE administration and muscle contraction on the expression of phosphorylated Akt (Ser473). Representative blots of phosphorylated Akt (Ser473) proteins corresponding to total Akt protein, followed by Ponceau S staining to verify equal protein loading. Values are presented as mean ± SD (*n* = 6); ^*∗*^*p* < 0.05.

**Figure 2:** Effects of LLE administration and muscle contraction on the expression of phosphorylated mTOR (Ser2448). Representative blots of phosphorylated mTOR (Ser2448) proteins corresponding to total mTOR protein, followed by Ponceau S staining to verify equal protein loading of proteins. Values are presented as mean ± SD (*n* = 6); ^*∗*^*p* < 0.05.

**Figure 3:** Effects of LLE administration and muscle contraction on the expression of phosphorylated p70S6K (Thr389). Representative blots of phosphorylated p70S6K (Thr389) protein corresponding to total p70S6K protein, followed by Ponceau S staining to verify equal protein loading. Values are presented as mean ± SD (*n* = 6); ^*∗*^*p* < 0.05.

## Data Availability

The data used to support the findings of this study are available from the corresponding author upon request.
